The article "Effect of lncRNA HULC knockdown on rat secreting pituitary adenoma GH3 cells" was retracted in 2020. Reason: concerns about the data.

# Effect of lncRNA HULC knockdown on rat secreting pituitary adenoma GH3 cells

**DOI:** 10.1590/1414-431X20197728

**Published:** 2019-04-15

**Authors:** Qiu Hong Rui, Jian Bo Ma, Yu Feng Liao, Jin Hua Dai, Zhen Yu Cai

**Affiliations:** 1 Department of Clinical Laboratory, HwaMei Hospital, University of Chinese Academy of Sciences (Ningbo No. 2 Hospital), Ningbo, Zhejiang, China; 2 Department of Pain Clinic, The First Affiliated Hospital of Xiamen University, Fujian Medical University, Xiamen, Fujian, China

**Keywords:** Secreting pituitary adenoma, LncRNA highly up-regulated in liver cancer (HULC), MicroRNA-130b, Forkhead box protein M1, PI3K/AKT/mTOR signaling pathway, JAK1/STAT3 signaling pathway

## Abstract

Pituitary adenoma is one of the most common tumors in the neuroendocrine system. This study investigated the effects of long non-coding RNAs (lncRNAs) highly up-regulated in liver cancer (HULC) on rat secreting pituitary adenoma GH3 cell viability, migration, invasion, apoptosis, and hormone secretion, as well as the underlying potential mechanisms. Cell transfection and qRT-PCR were used to change and measure the expression levels of HULC, miR-130b, and FOXM1. Cell viability, migration, invasion, and apoptosis were assessed using trypan blue staining assay, MTT assay, two-chamber transwell assay, Guava Nexin assay, and western blotting. The concentrations of prolactin (PRL) and growth hormone (GH) in culture supernatant of GH3 cells were assessed using ELISA. The targeting relationship between miR-130b and FOXM1 was verified using dual luciferase activity. Finally, the expression levels of key factors involved in PI3K/AKT/mTOR and JAK1/STAT3 pathways were evaluated using western blotting. We found that HULC was highly expressed in GH3 cells. Overexpression of HULC promoted GH3 cell viability, migration, invasion, PRL and GH secretion, as well as activated PI3K/AKT/mTOR and JAK1/STAT3 pathways. Knockdown of HULC had opposite effects and induced cell apoptosis. HULC negatively regulated the expression of miR-130b, and miR-130b participated in the effects of HULC on GH3 cells. FOXM1 was a target gene of miR-130b, which was involved in the regulation of GH3 cell viability, migration, invasion, and apoptosis, as well as PI3K/AKT/mTOR and JAK1/STAT3 pathways. In conclusion, HULC tumor-promoting roles in secreting pituitary adenoma might be via down-regulating miR-130b, up-regulating FOXM1, and activating PI3K/AKT/mTOR and JAK1/STAT3 pathways.

## Introduction

Pituitary adenoma, characterized by uncontrolled proliferation of pituitary gland cells, is one of the most common tumors in the neuroendocrine system (1,2). Pituitary adenomas can be divided into secreting and non-secreting pituitary adenomas (3). The clinical symptoms of secreting pituitary adenoma are dysfunction of the endocrine system, such as decreased libido, infertility, galactorrhea, and neurologic compression (like headaches and visual changes) (4). With the development of diagnostic and therapeutic methods, the 5-year survival rate of patients with secreting pituitary adenoma has increased in recent years (5,6). However, considering that the pathogenesis of this tumor is very complex (7,8), a clearer understanding of the process will be helpful for defining more effective diagnostic and therapeutic strategies.

The article "Effect of lncRNA HULC knockdown on rat secreting pituitary adenoma GH3 cells" was retracted in 2020. Reason: concerns about the data.

Long non-coding RNAs (lncRNAs) have been proved to exert critical regulatory roles in many biological processes, including cell proliferation, differentiation, and apoptosis (9). Aberrant expressions of lncRNAs have been linked to many human diseases, including secreting pituitary adenomas (10,11). As one kind of lncRNAs, highly up-regulated in liver cancer (HULC) is a key regulatory molecule that participates in the development and progression of hepatocellular carcinoma (12). Some studies in recent years demonstrated that HULC was also involved in the occurrence and development of other human cancers, such as osteosarcoma (13), epithelial ovarian carcinoma (14), bladder cancer (15), glioma (16), breast cancer (17), and chronic myeloid leukemia (18). However, there is no information available about the effects of HULC on pituitary adenoma, including secreting pituitary adenoma.

Similar to lncRNAs, microRNAs (miRNAs) also have important functions in the regulation of multiple cellular biological processes (19). Furthermore, lncRNAs can exert oncogenic or tumor suppressive roles by regulating the expressions of miRNAs in cells (20). miRNA-130b (miR-130b) has been shown to participate in cell proliferation and metastasis in many cancer cell lines (21). Leone et al. (22) reported that miR-130b was down-regulated in secreting pituitary adenoma.

Forkhead box protein M1 (FOXM1) is a typical cell proliferation-associated transcription factor, which stimulates cell proliferation by promoting S-phase and M-phase entries in cell cycle transition (23). Several reports provide evidence that the expression of FOXM1 is up-regulated in a variety of cancer cells (24). Many miRNAs can modulate the expression of FOXM1 in cancer cells (25,26). However, the role of FOXM1 in the regulation of secreting pituitary adenoma cell proliferation remains unclear.

Hence, in this research, we aimed to explore the effects of HULC on rat secreting pituitary adenoma GH3 cell line viability, migration, invasion, apoptosis, and hormone secretion, as well as miR-130b expression. The regulatory effect of miR-130b on FOXM1 expression in GH3 cells and regulatory roles of FOXM1 in GH3 cell viability, migration, invasion, and apoptosis were also investigated. Our findings will be helpful for further understanding the pathogenesis of secreting pituitary adenoma and provide potential diagnostic and therapeutic targets for secreting pituitary adenoma.

The article "Effect of lncRNA HULC knockdown on rat secreting pituitary adenoma GH3 cells" was retracted in 2020. Reason: concerns about the data.

## Material and Methods

### Cell lines

Rat secreting pituitary adenoma cell line GH3 and human embryonic kidney cell line HEK293 were obtained and authenticated by American Type Culture Collection (ATCC, USA, Cat. No. CCL-82.1 and CCL-1573). Cells were grown in Dulbecco's modified Eagle's medium (DMEM, Gibco, Life Technologies Corporation, USA) supplemented with 15% (v/v) fetal serum albumin (FBS, Hyclone, USA) and 1% (v/v) penicillin-streptomycin-glutamine (100X, Gibco, Life Technologies, USA). Cultures were maintained in a humidified incubator (Sanyo, Japan) at 37°C with 5% CO_2_. Transforming growth factor β (TGF-β, 10 ng/mL, Sigma-Aldrich, USA) was used as an inducer of cell migration and invasion.

### Isolation of rat pituitary primary cells

Three male Wistar rats (4 weeks, 124±12 g) were obtained from Shandong Laboratory Animal Center (China). Rats were acclimated in a temperature-controlled and specific pathogen-free environment for 4 days. Then, rats were sacrificed and the pituitary tissues were collected on ice. Subsequently, pituitary tissues were cut and trypsinized. The pituitary primary cells were collected by centrifugation (800 *g*, room temperature, 5 min).

### Cell transfection

Short-hairpin RNA directed against HULC and FOXM1 were ligated into U6/GFP/Neo plasmid (GenePharma Corporation, China) and referred to as sh-HULC and sh-FOXM1. The plasmid carrying a non-targeting sequence was used as negative control (NC) and referred to as sh-NC. The full-length sequences of HULC and FOXM1 were constructed in pcDNA3.1 plasmid (GenePharma Corporation) and referred to as pc-HULC and pc-FOXM1. The empty pcDNA3.1 plasmid acted as NC and referred to as pcDNA3.1. miR-130b mimic, miR-130b inhibitor and their NC were designed and synthesized by Life Technologies Corporation. The sequence of sh-HULC was 5′-AACCTCCAGAACTGTGATCCA-3′. The sequences of sh-FOXM1 were 5′-GCACAAGAACACTACTGTA-3′ (sense) and 5′-TACAGTAGTGTTCTTGTG C-3′ (antisense). The sequences of miR-130b mimic were 5′-ACUCUUUCCCUGUUGCACUACU-3′ (sense) and 5′-UAGUGCAACAGGGAAAGAGUUU-3′ (antisense). The sequence of miR-130b inhibitor was 5′-AGUAGUGCAACAGGGAAAGAGU-3′. The sequence of NC of miR-130b mimic and miR-130b inhibitor was 5′-UCACAACCUCCUAGAAAGAGUAGA-3′. Cell transfection was conducted using lipofetamine 3000 reagent (Invitrogen, USA) for 24 h. Transfection efficiencies of sh-HULC, pc-HULC, miR-130b mimic, and miR-130b inhibitor were verified using quantitative reverse transcription (qRT-PCR). Transfection efficiencies of pc-FOXM1 and sh-FOXM1 were verified using qRT-PCR and western blotting.

The article "Effect of lncRNA HULC knockdown on rat secreting pituitary adenoma GH3 cells" was retracted in 2020. Reason: concerns about the data.

### qRT-PCR

qRT-PCR was performed to detect the expression levels of HULC, miR-130b, and FOXM1 in GH3 cells after relevant transfection. Briefly, total RNAs in GH3 cells were isolated using TRIzol^TM^ Plus RNA Purification kit (Invitrogen). The cDNA was reversely transcribed using high capacity cDNA reverse transcription kit (Applied Biosystems, USA). Then, the expression levels of HULC and FOXM1 were measured using TaqMan^TM^ real-time PCR master mix (Applied Biosystems). The expression level of miR-130b was measured using TaqMan^TM^ non-coding RNA assay (Applied Biosystems). The expression levels of β-actin and U6 acted as endogenous controls. Data were quantified by 2^−△△Ct^ method (27). The primer sequences of HULC were 5′-ACCTCCAGAACTGTGATCCAAAATG-3′ (sense) and 5′-TCTTGCTTGATGCTTTGGTCTG-3′ (antisense). The primer sequence of miR-130b was 5′-ACACTCCAGCTGGGACTCTTTCCCTGTTGC-3′. The primer sequences of FOXM1 were 5′-TCCAGAGCATCATCACAGCG-3′ (sense) and 5′-TGCTCCAGGTGACAATTCTCC-3′ (antisense). The primer sequences of β-actin were 5′-GAGAGGGAAATCGTGCGTGAC-3′ (sense) and 5′-CATCTGCTGGAAGGTGGACA-3′ (antisense). The primer sequences of U6 were 5′-CAAATTCGTGAAGCGTT-3′ (sense) and 5′-TGGTGTCGTGGAGTCG-3′ (antisense).

### Cell viability assay

Cell viability was assessed using trypan blue staining assay kit (Beyotime Biotechnology, China) and 3-(4,5-dimethylthiazol-2-yl)-2,5-diphenyltertrazolium bromide tetrazolium (MTT) assay (Sigma-Aldrich). For trypan blue staining, after relevant transfection, GH3 cells were seeded into a 6-well plate (Thermo Fisher Scientific, USA) with 1 × 10^5^ cells per well and cultured at 37°C for 24 h. Then, cells were collected, washed with phosphate-buffered saline (PBS), stained using the kit solution, and counted under a microscope (Nikon, Japan). Cell viability (%) was calculated by number of viable cells / number of total cells × 100%.

For the MTT assay, after relevant transfection, GH3 cells were seeded into a 96-well plate (Thermo Fisher Scientific) with 1 × 10^4^ cells per well and cultured at 37°C for 24 h. Then, 20 μL MTT solution (2.5 mg/mL in PBS) was added into the medium of each well and the plate was incubated at 37°C for 4 h. Subsequently, the MTT mixture was removed and 150 μL dimethyl sulfoxide (DMSO) was added to dissolve formazan. After that, the plate was agitated on a shaker for 15 min. The absorbance of each well at 570 nm was recorded using a microplate reader (Bio-Tek Instrument, USA).

The article "Effect of lncRNA HULC knockdown on rat secreting pituitary adenoma GH3 cells" was retracted in 2020. Reason: concerns about the data.

### Cell migration and invasion assay

Cell migration was determined using a modified two-chamber transwell assay (Corning Incorporated, USA). Briefly, after relevant transfection, 1 × 10^3^ GH3 cells were suspended in 200 μL serum free-DMEM and added into the upper chamber. Complete DMEM (600 μL) was added into the lower chamber. After incubation at 37°C for 48 h, cells were immediately fixed with 4% paraformaldehyde solution (Beyotime Biotechnology, China). Then, non-migrated cells in the upper chamber were removed carefully using a cotton swab and migrated cells in the lower chamber were counted under a microscope (Nikon, Japan). Cell migration (%) was calculated by average number of migrated cells in transfection group / average number of migrated cells in control group × 100%.

Cell invasion was evaluated similarly with cell migration, except that the transwell membrane was pre-incubated using Matrigel (BD Biosciences, USA). Cell invasion (%) was calculated by average number of invaded cells in transfection group / average number of invaded cells in control group × 100%.

### Cell apoptosis assay

Guava Nexin assay (Millipore Billerica, USA) was used to detect the apoptosis of GH3 cells. Briefly, after relevant transfection, GH3 cells were seeded into a 6-well plate with 1 × 10^5^ cells per well and cultured at 37°C for 24 h. Then, cells were collected, washed with PBS, stained using the kit solution, and subjected to flow cytometry analysis (Guava easyCyte 8HT, Millipore Billerica, USA). Data were analyzed using FCS Express software (De Novo software, USA).

### Enzyme linked immunosorbent assay (ELISA)

ELISA was conducted to measure the concentrations of prolactin (PRL) and growth hormone (GH) in culture supernatant of GH3 cells. Briefly, after relevant transfection, GH3 cells were seeded into a 6-well plate with 1 × 10^5^ cells per well and cultured at 37°C for 24 h. Then, the cell supernatant of each group was collected and concentrations of PRL and GH were measured using rat PRL ELISA kit and rat GH ELISA kit (Invitrogen), respectively.

### Dual luciferase activity assay

The 3′ untranslated region (UTR, 2257-3049 bp) fragment of FOXM1, containing the predicted miR-130b binding site, was amplified by PCR and constructed in pmirGLO vector (Promega, USA) to form FOXM1-wild type (FOXM1-wt). To mutate the predicted miR-130b binding site, the predicted binding site was replaced, amplified, and constructed in pmirGLO vector to form FOXM1-mutated type (FOXM1-mt). The sequence of FOXM1-wt was 5′-CAAAGGCAAUGGUGAAAAGAGAU-3′ and the sequence of FOXM1-mt was 5′-CAAAGGCAAUGGUGACAGUUAAU-3′. Then, miR-130b mimic and reporter vectors were transfected into HEK293 cells simultaneously. The relative luciferase activity was detected using dual-luciferase reporter assay system (Promega).

The article "Effect of lncRNA HULC knockdown on rat secreting pituitary adenoma GH3 cells" was retracted in 2020. Reason: concerns about the data.

### Western blotting

Western blotting was performed as previously described (28). Briefly, total proteins in GH3 cells were isolated using RIPA lysis buffer (Beyotime Biotechnology, China) containing protease inhibitors (Roche, Switzerland) and quantified using BCA protein assay kit (Beyotime Biotechnology). Then, proteins in equal concentrations were electrophoresed in polyacrylamide gels and transferred onto nitrocellulose membranes (Millipore, USA). All primary antibodies were prepared in 1% bovine serum albumin (BSA, Beyotime Biotechnology) solution at a dilution of 1:1000. After incubation with 5% BSA at room temperature for 1 h, the membranes were incubated with primary antibodies against E-cadherin (ab1416), N-cadherin (ab18203), Vimentin (ab137321), Snail (ab53519), poly ADP-ribose polymerase (PARP, ab32138), cleaved-PARP (ab32064), Pro-caspase 3 (ab4051), cleaved-caspase 3 (ab49822), Pro-caspase 9 (ab2013), FOXM1 (ab180710), p-phosphatidylinositol 3-kinase (PI3K, ab182651), t-PI3K (ab191606), p-protein kinase 3 (AKT, 38449), t-AKT (ab8805), p-mammalian target of rapamycin (mTOR, ab137133), t-mTOR (ab2732), β-actin (ab8226, Abcam Biotechnology, USA), p-janus kinase 1 (JAK1, #74129), t-JAK1 (#3344), p-signal transducing activator of transcription 3 (STAT3, #9145), t-STAT3 (#9139), and Cleaved-caspase 9 (#9507, Cell Signaling Technology, USA) at 4°C overnight. Then, the membranes were incubated with goat anti-rabbit (or anti-mouse) IgG H&L (HRP) secondary antibodies (ab205718, ab205719, Abcam Biotechnology) for 1.5 h at room temperature. Followed by adding 200 μL Immobilon western chemiluminescent HRP substrate (Millipore) to the surfaces of membranes, the signals of proteins were captured using Bio-Rad ChemiDoc^TM^ XRS system (Bio-Rad Laboratories, USA). Intensities of bands were quantified using Image Lab^TM^ software (Bio-Rad Laboratories).

### Statistical analysis

All experiments were conducted at least three times. Results of multiple experiments are reported as means±SD. Graphpad 6.0 software (Graphpad, USA) was used for statistical analysis. P values were calculated using one-way analysis of variance (ANOVA). Statistically significant differences were set at P<0.05.

## Results

### HULC was highly expressed in GH3 cells

Firstly, we detected the expression level of HULC in rat pituitary primary cells and rat secreting pituitary adenoma GH3 cells. The results in Figure 1 show that HULC was highly expressed in GH3 cells, compared to rat pituitary primary cells (P<0.01). This finding suggested that HULC might exert oncogenic roles in secreting pituitary adenoma.

The article "Effect of lncRNA HULC knockdown on rat secreting pituitary adenoma GH3 cells" was retracted in 2020. Reason: concerns about the data.

**Figure 1.** Highly up-regulated in liver cancer (HULC) was highly expressed in GH3 cells. The expression level of HULC in rat pituitary primary cells (PPC) and rat secreting pituitary adenoma GH3 cells was detected using qRT-PCR. Data are reported as means±SD. **P<0.01 (ANOVA).

### HULC exerted oncogenic roles in GH3 cells

Figure 2A shows that the expression level of HULC was significantly decreased after sh-HULC transfection (P<0.01) and increased after pc-HULC transfection (P<0.01). Figure 2B–E shows that knockdown of HULC remarkably suppressed the viability, migration, and invasion of GH3 cells (P<0.05 or P<0.01). On the contrary, overexpression of HULC had opposite effects, which notably enhanced the viability, migration, and invasion of GH3 cells (P<0.05 or P<0.01). Figure 2F shows that TGF-β treatment promoted GH3 cell migration and invasion via reducing the expression level of E-cadherin and enhancing the expression levels of N-cadherin, vimentin, and Snail. Compared to the TGF-β single treatment group, the expression level of E-cadherin was increased, and the expression levels of N-cadherin, vimentin, and Snail were decreased in TGF-β treatment+sh-HULC transfection group. pc-HULC transfection had opposite effects.

**Figure 2.** Highly up-regulated in liver cancer (HULC) exerted oncogenic roles in GH3 cells. After sh-HULC or pc-HULC transfection, **A**, the expression of HULC in GH3 cells, **B**–**E**, the viability, migration, and invasion of GH3 cells, **F**, the expression levels of E-cadherin, N-cadherin, vimentin, and snail in GH3 cells, **G**, the apoptosis of GH3 cells, **H**, the expression levels of PARP, cleaved-PARP, pro-caspase 3, cleaved-caspase 3, pro-caspase 9, and cleaved-caspase 9 in GH3 cells, and **I** and **J**, the concentration of prolactin (PRL) and growth hormone (GH) in culture supernatant of GH3 cells were assessed using qRT-PCR, trypan blue staining assay, MTT assay, two-chamber transwell assay, Guava Nexin assay, western blotting, and ELISA. NC: negative control; TGF-β: transforming growth factor β; PARP: poly ADP-ribose polymerase. Data are reported as means±SD. *P<0.05, **P<0.01, ^#^P<0.05, ^##^P<0.01 compared to pcDNA3.1 group (ANOVA).

Moreover, the results of Figure 2G show that HULC knockdown markedly induced GH3 cell apoptosis (P<0.01). Western blotting showed that the expression levels of cleaved-PARP, cleaved-caspase 3, and cleaved-caspase 9 in GH3 cells were all increased after HULC knockdown (Figure 2H). Furthermore, Figure 2I and J show that HULC knockdown notably reduced the concentrations of PRL and GH in culture supernatant of GH3 cells (P<0.05). On the contrary, overexpression of HULC dramatically enhanced the concentrations of PRL and GH in culture supernatant of GH3 cells (P<0.05). Taken together, these results suggested that HULC exerted oncogenic roles in GH3 cells. Knockdown of HULC inhibited GH3 cell viability, migration, invasion, and hormone secretion, but promoted cell apoptosis.

The article "Effect of lncRNA HULC knockdown on rat secreting pituitary adenoma GH3 cells" was retracted in 2020. Reason: concerns about the data.

### HULC negatively regulated the expression of miR-130b in GH3 cells

The expression level of miR-130b in GH3 cells after HULC knockdown or overexpression was measured using qRT-PCR. As presented in Figure 3, HULC knockdown enhanced the expression level of miR-130b (P<0.01) and overexpression of HULC significantly reduced the expression level of miR-130b in GH3 cells (P<0.05). This finding indicated that HULC negatively regulated the expression of miR-130b in GH3 cells and implied that miR-130b might be involved in the effects of HULC on GH3 cells.

**Figure 3.** Highly up-regulated in liver cancer (HULC) negatively regulated the expression of miR-130b in GH3 cells. After sh-HULC or pc-HULC transfection, the expression level of miR-130b in GH3 cells was detected using qRT-PCR. miR-130b: MicroRNA-130b; NC: negative control. Data are reported as means±SD. *P<0.05; **P<0.01 (ANOVA).

### miR-130b participated in the effects of HULC on GH3 cell viability, migration, invasion, and apoptosis

The expression level of miR-130b in GH3 cells was increased after miR-130b mimic transfection (P<0.01) and decreased after miR-130b inhibitor transfection (P<0.01, Figure 4A). The results of Figure 4B–D show that HULC knockdown-induced GH3 cell viability, migration, and invasion inhibition were markedly aggravated by miR-130b overexpression (P<0.05) and inhibited by miR-130b suppression (P<0.05). Moreover, Figure 4E shows that HULC knockdown-induced GH3 cell apoptosis enhancement was also aggravated by miR-130b overexpression (P<0.05) and inhibited by miR-130b suppression (P<0.05). Compared to the sh-HULC+NC group, the expression levels of cleaved-PARP, cleaved-caspase 3, and cleaved-caspase 9 in GH3 cells were increased in sh-HULC+miR-130b mimic group and decreased in sh-HULC+miR-130b inhibitor group (Figure 4F). These results suggested that knockdown of HULC inhibited GH3 cell viability, migration, and invasion, as well as induced GH3 cell apoptosis, which might be via up-regulating miR-130b.

**Figure 4.** miR-130b participated in the effects of highly up-regulated in liver cancer (HULC) on GH3 cell viability, migration, invasion, and apoptosis. **A**, Expression of miR-130b in GH3 cells after miR-130b mimic or miR-130b inhibitor transfection was measured using qRT-PCR. After sh-HULC and/or miR-130b mimic (inhibitor) transfection, **B**–**E**, the viability, migration, invasion, and apoptosis of GH3 cells, and **F**, the expression levels of PARP, cleaved-PARP, pro-caspase 3, cleaved-caspase 3, pro-caspase 9, and cleaved-caspase 9 in GH3 cells were assessed using trypan blue staining assay, two-chamber transwell assay, Guava Nexin assay, and western blotting. miR-130b: microRNA-130b; NC: negative control; PARP: poly ADP-ribose polymerase. Data are reported as means±SD.*P<0.05, **P<0.01 (ANOVA).

The article "Effect of lncRNA HULC knockdown on rat secreting pituitary adenoma GH3 cells" was retracted in 2020. Reason: concerns about the data.

### FOXM1 was target gene of miR-130b in GH3 cells

The mRNA and protein expression levels of FOXM1 in GH3 cells after miR-130b mimic or miR-130b inhibitor transfection were detected in this research. As displayed in Figure 5A, the mRNA and protein expression levels of FOXM1 in GH3 cells were reduced after miR-130b mimic transfection (P<0.05 in mRNA level) and enhanced after miR-130b inhibitor transfection (P<0.01 in mRNA level). Figure 5B shows that the relative luciferase activity was notably decreased after co-transfection with miR-130b mimic and FOXM1-wt (P<0.05). The potential binding sequence between miR-130b and 3′UTR of FOXM1 is shown in Figure 5C. These findings indicated that miR-130b negatively regulated the expression of FOXM1 and FOXM1 was a target gene of miR-130b in GH3 cells.

**Figure 5.** FOXM1 was a target gene of miR-130b in GH3 cells. **A**, The mRNA and protein expression levels of FOXM1 in GH3 cells after miR-130b mimic or miR-130b inhibitor transfection were determined using qRT-PCR and western blotting. **B**, Relative luciferase activities were detected after co-transfection with miR-130b mimic and FOXM1-wt (FOXM1-mt). **C**, Bioinformatics analysis was used to predict the potential binding sequence between miR-130b and 3′UTR of FOXM1. miR-130b: microRNA-130b; FOXM1: forkhead box protein M1; NC: negative control; wt: wild type; mt: mutated type. Data are reported as means±SD.*P<0.05; **P<0.01 (ANOVA).

### Overexpression of FOXM1 promoted the viability, migration, and invasion of GH3 cells

The results in Figure 6A show that pc-FOXM1 transfection increased the mRNA and protein levels of FOXM1 (P<0.01 in mRNA level) and sh-FOXM1 transfection decreased the mRNA and protein levels of FOXM1 in GH3 cells (P<0.01 in mRNA level). Figure 6B–D shows that the viability, migration, and invasion of GH3 cells were remarkably enhanced after pc-FOXM1 transfection (P<0.05 or P<0.01) and reduced after sh-FOXM1 transfection (P<0.05 or P<0.01). In addition, Figure 6E shows that sh-FOXM1 transfection induced GH3 cell apoptosis (P<0.01). Similar results were found by western blotting, which illustrated that the expression levels of cleaved-PARP, cleaved-caspase 3, and cleaved-caspase 9 in GH3 cells were all increased in sh-FOXM1 transfection group (Figure 6F). These above findings indicated that FOXM1 also played oncogenic roles in GH3 cells.

The article "Effect of lncRNA HULC knockdown on rat secreting pituitary adenoma GH3 cells" was retracted in 2020. Reason: concerns about the data.

**Figure 6.** After pc-FOXM1 or sh-FOXM1 transfection, **A**, the mRNA and protein levels of FOXM1, **B**–**E**, the viability, migration, invasion, and apoptosis of GH3 cells, and **F**, the expression levels of PARP, cleaved-PARP, pro-caspase 3, cleaved-caspase 3, pro-caspase 9, and cleaved-caspase 9 in GH3 cells were assessed using qRT-PCR, western blotting, trypan blue staining assay, two-chamber transwell assay, and Guava Nexin assay. FOXM1: Forkhead box protein M1; NC: negative control; PARP: poly ADP-ribose polymerase. Data are reported as means±SD. *P<0.05; **P<0.01 (ANOVA).

### HULC and FOXM1 participated in the regulation of PI3K/AKT/mTOR and JAK1/STAT3 pathways in GH3 cells

Figure 7A and B show that overexpression of HULC activated PI3K/AKT/mTOR and JAK/STAT3 pathways via up-regulating the expression rates of phosphate/total-PI3K (p/t-PIEK), p/t-AKT, p/t-mTOR, p/t-JAK1, and p/t-STAT3 in GH3 cells (P<0.01). Suppression of HULC had opposite effects, which inactivated PI3K/AKT/mTOR and JAK/STAT3 pathways via down-regulating the expression rates of p/t-PI3K, p/t-AKT, p/t-mTOR, p/t-JAK1, and p/t-STAT3 in GH3 cells (P<0.01). Moreover, Figure 7C and D displays that FOXM1 overexpression activated PI3K/AKT/mTOR and JAK/STAT3 pathways by enhancing the expression rates of p/t-PI3K, p/t-AKT, p/t-mTOR, p/t-JAK1, and p/t-STAT3 (P<0.05 or P<0.01). Suppression of FOXM1 inactivated PI3K/AKT/mTOR and JAK/STAT3 pathways by reducing the expression rates of p/t-PI3K, p/t-AKT, p/t-mTOR, p/t-JAK1, and p/t-STAT3 (P<0.05). Taken together, these findings suggested that HULC and FOXM1 were involved in the regulation of PI3K/AKT/mTOR and JAK1/STAT3 pathways in GH3 cells and exerted oncogenic roles in GH3 cells, which might be via activating PI3K/AKT/mTOR and JAK1/STAT3 pathways.

**Figure 7.** Overexpression of FOXM1 activated PI3K/AKT/mTOR and JAK1/STAT3 pathways in GH3 cells. (**A** and **B**) The expression levels of p-PI3K, t-PI3K, p-AKT, t-AKT, p-mTOR, t-mTOR, p-JAK1, t-JAK1, p-STAT3, and t-STAT3 in GH3 cells after pc-HULC or sh-HULC transfection were evaluated using western blotting. (**C** and **D**) The expression levels of the same proteins in GH3 cells after pc-FOXM1 or sh-FOXM1 transfection were evaluated using western blotting. HULC: Highly up-regulated in liver cancer; FOXM1: forkhead box protein M1; NC: negative control; PI3K: phosphatidylinositol 3-kinase; AKT: protein kinase 3; mTOR: mammalian target of rapamycin; JAK1: janus kinase 1; STAT3: signal transducing activator of transcription 3. Data are reported as means±SD. *P<0.05; **P<0.01 (ANOVA).

The article "Effect of lncRNA HULC knockdown on rat secreting pituitary adenoma GH3 cells" was retracted in 2020. Reason: concerns about the data.

## Discussion

Pituitary adenoma comprises approximately 10–15% of all tumors in the central nervous system (2,3,29). lncRNAs and miRNAs can function as oncogenes or tumor suppressors, and exert critical regulatory roles in the carcinogenesis of multiple cancers, including pituitary adenoma (19). In this study, we revealed that HULC had a higher expression level in secreting pituitary adenoma GH3 cells, compared to rat pituitary primary cells. Overexpression of HULC significantly promoted the viability, migration, invasion, and hormone secretion of GH3 cells, as well as down-regulated the expression of miR-130b. Knockdown of HULC had opposite effects and induced GH3 cell apoptosis. Furthermore, we also found that FOXM1 was a target gene of miR-130b in GH3 cells and participated in the regulation of GH3 cell viability, migration, invasion, and apoptosis, as well as PI3K/AKT/mTOR and JAK1/STAT3 signaling pathways.

lncRNAs do not encode proteins, but play important roles in the regulation of gene expression in cells (9,30). Numerous studies have proved the oncogenic roles of HULC in cancer cells by their contribution on cancer cell proliferation and metastasis (13,15). For example, Chen et al. (14) reported that overexpression of HULC promoted proliferation, migration, and invasion of epithelial ovarian carcinoma cells. Matouk et al. (31) indicated that HULC was related to metastasis of colorectal carcinomas. Our results were consistent with previous studies.

Abnormal hormone secretion is one of the major complications of secreting pituitary adenomas (32). As a rat secreting pituitary adenoma cell line, GH3 can also secret PRL and GH (33). Therefore, we also assessed the PRL and GH levels in culture supernatant of GH3 cells after HULC overexpression or knockdown. Taken together, our results revealed the critical roles of HULC in regulating rat secreting pituitary adenoma cell proliferation, metastasis, and hormone secretion.

One of the most important findings in this research was that HULC negatively regulated the expression of miR-130b in GH3 cells. Reports have proved that miRNAs are involved in the regulation of intracellular gene expression at the post-transcriptional level (19,34). miR-130b has been demonstrated to be down-regulated in pituitary adenomas cells, including secreting pituitary adenoma (22). The findings of the present study suggested that HULC exerted oncogenic roles in rat secreting pituitary adenoma GH3 cells at least in part by down-regulating miR-130b.

As a typical cell proliferation-associated transcription factor, FOXM1 plays important roles in regulating cell proliferation (35). Moreover, FOXM1 has a high expression level in many human cancer cells (24,36). In this study, we revealed that FOXM1 was a target gene of miR-130b in GH3 cells. The findings indicated that miR-130b participated in the effects of HULC on GH3 cells, which might be through regulating FOXM1.

The article "Effect of lncRNA HULC knockdown on rat secreting pituitary adenoma GH3 cells" was retracted in 2020. Reason: concerns about the data.

PI3K/AKT/mTOR and JAK1/STAT3 signaling pathways play critical roles in the regulation of multiple cell functions, such as cell proliferation, cell invasion, and cell apoptosis (37,38). Tian et al. (39) proved that miR-361-5p inhibited chemo-resistance of gastric cancer cells by targeting FOXM1 and PI3K/AKT/mTOR signaling pathway. Buslei et al. (40) reported that the activation of JAK1/STAT3 signaling pathway contributed to the development of pituitary adenoma. Thus, in this research, we also analyzed the effects of HULC and FOXM1 on the activation of PI3K/AKT/mTOR and JAK1/STAT3 pathways in GH3 cells. The results suggested that HULC exerted oncogenic roles in GH3 cells, which might be via down-regulating miR-130b, up-regulating FOXM1, and then activating PI3K/AKT/mTOR and JAK1/STAT3 pathways.

In summary, our research verified the oncogenic roles of HULC in rat secreting pituitary adenoma GH3 cells. This study contributes to the further understanding of the pathogenesis of secreting pituitary adenomas and is helpful for defining potential diagnostic and therapeutic targets.
